# Visualization Display System of Gannan Hakka Paper-Cut Works Based on Computer Graphics Algorithm

**DOI:** 10.1155/2022/2419689

**Published:** 2022-03-24

**Authors:** Xingping Li

**Affiliations:** Ganzhou Teachers College, Ganzhou, Jiangxi 341000, China

## Abstract

Today, computer graphics and graphic image processing techniques have been widely used in daily life and industrial production. Due to the development of computers, computer graphics has brought more convenience to our daily life. In order to give full play to the value of computers, this paper takes the Hakka paper-cut art with local characteristics as the starting point, first of all its development history, artistic characteristics, compositional forms, expression techniques, cultural connotations, Hakka paper-cut patterns, and the symbolic meaning of folk customs, and then we design a visualization system for the paper-cut works of Gannan Hakka based on computer graphics. In addition, the system provides a solution for the integration of Gannan Hakka paper-cut art and Jiangxi native product packaging design and provides a reference for the theory and practice of modern native product packaging design.

## 1. Introduction

Computer graphics (CG) is a scientific area that studies the representation, production, processing, and display of visual images using computer technology. The development of computer graphics has spanned more than 40 years, and it has grown to become one of the most active disciplines of computer science, with widespread application. The scanning transformation of straight lines, the scanning transformation of circular arcs, the scanning transformation of polygons and area filling, character representation, area cropping, antiwalking, shading, and other aspects of computer graphics research are among the most important topics in the field. In most domestic institutions of higher education, the course of computer graphics is currently provided as part of the related majors in the majority of schools. As part of the computer graphics curriculum, students will learn how to generate graphics and process them using algorithms. The course will be difficult because students will have to understand and master algorithms. The development of computer graphics visualization teaching platforms is an urgent requirement for computer graphics education [1–8].

The background of the information age is constantly improving, and the impact of information technology on daily life and work is also becoming more and more profound. As a result, computer graphics and graphic image processing technology have become an indispensable part of our daily work and personal lives. The effective application of computer graphics and graphic image processing technology can significantly improve the level of mass graphic image processing when compared to traditional image processing modes, thereby improving the design efficiency and performance of various fields and thus significantly enriching the cultural and entertainment lives of the general public. Consequently, computer graphics and visual image processing techniques are now widely used in a wide range of industries, including medicine [9].

Based on the paper-cut pattern library, researchers have constructed several auxiliary design systems that can express the meaning of paper-cut patterns, such as the computer-aided paper-cut generation method for animal patterns [10, 11]. In addition, Talked Sukumar et al. [12] developed a CAD system for synthesizing kirigami patterns. Sun et al. [13] proposed a paper-cut pattern simulation method that supports tools such as folding, cutting, and unfolding.

In computer graphics, geometric elements such as points, lines, surfaces, and bodies, as well as nongeometric properties such as grayscale colors, line forms, and line widths, are used to create visual effects. Among the many types of content that computer graphics encompasses, there are graphics hardware; solid modeling; graphics interaction techniques; computer visualization, which includes natural scene simulation; computer animation; and virtual reality, among other things [14–16].

A thread is a collection of instructions or a particular section of a program, which can be run independently inside the program but must be contained within a dependent process and can only access resources and information that are held by the dependent process. It might also be interpreted as the environment in which the code is executed. Schwab et al. [17] developed a paper-cut tool that can engrave patterns on the surface of 3D models, and Aili [18] proposed a computer-generated method of paper-cut style flowing animation. The establishment and use of the pattern library greatly facilitate the expression of the cultural meaning of paper-cutting, but the existing methods focus on the interactive design of patterns and lack in-depth analysis of its spatial structure [19].

For the sake of this discussion, threads can be considered lightweight processes that are responsible for performing various tasks within a single program. Most of the time, the operating system is in charge of the scheduling and execution of numerous threads simultaneously. Another program, or process, must have a main thread, which serves as the entry point for executing code and initiating the program's execution. Multithreading is a programming mechanism that allows the concurrent execution of many instruction streams in a program, each of which is referred to as a thread, which are independent of one another but still being able to communicate with one another [20, 21]. Multithreading is a technique for making numerous threads work in parallel to complete multiple tasks at the same time in order to boost the overall efficiency of the system.

With the rapid development of the product economy, regional specialties with distinct regional characteristics and personality characteristics gradually demonstrate obvious advantages and gradually establish themselves as significant support for the development of the regional economy and the driving force for the development of other industries. At the moment, one of the most pressing issues is how to package local specialties that have distinct regional cultural qualities and connotations while also maximizing their economic value. This is a difficult problem to tackle.

In order to construct a suitable digital model, this paper proposes a visualization system of Gannan Hakka paper-cut works based on computer graphics algorithms and proposes a bottom-up spatial analysis method of paper-cut construction patterns. The method can extract the boundary pixels of the scanned image of kirigami, obtain each kirigami pattern through preprocessing such as denoising and vectorization, build element layers, and cluster the kirigami patterns according to the similarity to obtain similar layers and then detect the same class. Spatial distribution pattern of kirigami patterns so as to identify the paper-cut pattern and establish the pattern layer. Finally, the paper-cut works of Gannan Hakka can be classified, displayed, and automatically classified.

The research route of the dissertation includes the following steps.

The first section introduces the main content of the full text, the second section introduces computer graphics, the third section introduces the application of computer graphics, the fourth section introduces digital modeling and visual presentation of paper cuttings, and the fifth section summarizes the full text.

## 2. Computer Graphics

### 2.1. Overview of Computer Graphics and Graphic Image Processing Techniques

- Computer graphics is a branch of computer science that deals with visual representations of information.
- When two- or three-dimensional visuals are transformed into a grid within a computer monitor, computer graphics is defined as the study of applying mathematical methods to achieve this transformation. When computer algorithms and related information techniques are used to execute effective calculations, graphics processing, and transformation and to properly actualize the information processing of graphics with the support of computer hardware, the study of computer graphics is possible. Taking virtual reality technology as an example, it is a technological advancement that makes use of computer information technology to create and process geometric shapes in order to provide a realistic experience of things. A significant impact has been made by the development of computer graphics on the design work in various fields, particularly in light of the rapid development of the market economy. The application of computer graphics can help to improve the overall product and service quality, as well as more effectively meeting the demands of consumers through the use of intuitive design graphics and images.
- Computer-aided design and production technology.
- With the use of computer software, graphic image processing technology is used to develop and optimize graphic pictures, which then collaborate with one another with the help of computer system software and hardware, according to the appropriate processing needs. CAM, CAD, CAI, and other software techniques are often employed in the processing process, while the hardware needs to be realized with the help of various image processors, such as pictures, keyboards, CPUs, and other similar devices. With the help of this software and hardware, as well as the level of computer processing, it is possible to effectively achieve geometric deformation processing, which allows for the efficient performance of recovery, segmentation, and other operations, as well as the achievement of the most anticipated image processing effect from the start.

### 2.2. Practical Applications of Computer Graphics and Graphic Image Processing Techniques

1. Industrial applications of the technology.
2. The use of computer graphics and image processing technology in industrial production is becoming increasingly common. Computer-aided design (CAD) and manufacturing (CAM) software are frequently used in the design and construction of aircraft and automobiles, huge machinery, and clothes, among other things. Examples include the design and production of automobiles, where manufacturers use computer-aided design (CAD) systems to create the structure and appearance of new cars, then analyze and adjust the design graphics to significantly improve their appearance, and finally employ computer-aided assembly (CA) systems to significantly optimize the structure of new cars in order to achieve the best design while reducing production costs. In addition, computer graphics and graphic image processing techniques are frequently utilized in the construction business and are mostly used in the production of engineering drawings, 3D modeling of buildings, and other related tasks. The introduction of graphics and graphic image processing techniques to modeling processing can result in a more intuitive display of the full building structure, resulting in a more image-specific construction overall.
3. Commercial applications in a variety of fields.
4. Computer graphics and graphic image processing techniques have become more widely used in the commercial field as the social economy has progressed, specifically in the production of computer and mobile games, advertising design, animation production, film and television special effects production, and a variety of other fields. This commercial application of computer graphics and graphic image processing technology takes the form of computer animation in most cases. For example, the animated effects we see in advertisements, commercial advertising campaigns, and LED electronic screen advertisements are all examples of computer animation. This also reflects the close connection between computer graphics and graphic image processing technology and real life.
5. Application in the realm of artistic expression.
6. In recent years, the continuous development of computer graphics and graphic image processing technology has had an impact and influence on the art field, and many artists are now using computer drawing software and a touch panel to create computer paintings, which is a departure from the traditional painting mode. The use of these hardware devices to create art paintings allows us to make effective use of the various functions in the drawing software to process the details and adjust the colors accordingly, thereby reducing the restrictions on the materials available for painting creation and enriching and expanding the space available for art painting creation effectively. Additionally, 3D modeling software may be used efficiently in the design and fabrication of sculptures, which helps designers to better create and conceptualize their works, boosting the aesthetic expression of sculptures even further.
7. In the fields of environmental protection, meteorology, and molecular biology, the technology has found use.
8. There is a great deal of complicated scientific computer information in the domains of environmental protection, meteorology, and molecular biology, and it takes a long time to process this information. When computer graphics and image processing technology are properly applied, it can effectively realize the visualization of data information, including complex and difficult to understand data information, with intuitive graphics and image presentation, allowing researchers to use it for research and analysis purposes. Examples include the process of meteorological observation, whereby a large number of pieces of meteorological data information can be effectively organized and then intuitively displayed using satellite cloud maps, allowing for reasonable predictions and analysis of meteorological changes. Computer graphics and graphic image processing technology can be used to effectively organize and display the relevant data. Because of this technique, researchers can effectively organize complex biological research data into molecular structure diagrams so that they may study and interpret the data in intuitive visuals, which is very useful for complex biological research.
9. The use of the technology in the field of multimedia.
10. Additionally, computer graphics and graphic image processing techniques are employed in the field of multimedia, with their application primarily referring to the efficient operation, generation, storage, and communication of multimedia information through the use of computer control, also known as a grassroots information system. These techniques enable the processing of graphics, video, photos, and other pieces of information included in multimedia, allowing for the diversification of multimedia graphics information. For example, with the help of computer graphics and graphic image processing technology, it is possible to enrich the content of multimedia teaching materials by including animation, audio, and other means of mobilizing the students' sensory perceptions, thereby improving the overall effectiveness of the use of multimedia teaching materials.

## 3. Applications of Computer Graphics

### 3.1. Imagery Beauty

The Hakka are a community with a rich traditional culture, and the Hakka people of the Central Plains have demonstrated exceptional inclusivity in the compatibility and transmission of culture and art across generations. The craft of paper-cutting has a long history among the Hakka people of Gannan, and it demonstrates particular regional cultural characteristics. For example, the paper-cutting works “Five Lucky Men,” “Seven Lucky Stars,” and “Eight Immortals Crossing the Sea” in Ningdu are not constrained by real or objective limits, and they accurately portray the imagination and expression of the Hakka people in their entirety. They are a beautiful representation of the Hakka people's inventiveness and expressiveness, and they exhibit a wonderful aesthetic style and cultural significance.

### 3.2. The Appeal of the Subject Matter

It is beautiful in its ruggedness and simplicity, and it is rich in subject matter and emotion. The paper-cutting of the Hakka people of Gannan is rich in subject matter and emotion, and it is simple in style. Houses, landscapes, characters, folklore, and labor scenes are common subjects for paper-cutting, which show the traits of Hakka people's hard work, purity and simplicity, solidarity, and love of life, together with significant regional cultural characteristics (see Figures 1 and 2).

When it comes to the symbolic expression of peace, luck, and happiness, the Hakka paper-cutting patterns seen in Gannan are particularly noteworthy. Hakka people will decorate their rooms, halls, and courtyards with auspiciousness and joy during some folk festivals and celebrations in order to express their good wishes for future life. They will also place paper cutouts with corresponding themes on their doors, windows, and utensils to demonstrate their participation in the celebration. Paper-cutting works with auspicious patterns such as the magpie, lotus, longevity peach, and fortune characters created by paper-cutting artists are covered on the table of sacrificial offerings in some traditional rituals, which serve as both decorative elements and vehicles for conveying people's good wishes at the same time. In the Hakka wedding tradition, large red “Shao,” “Fu,” “Lu,” “Cai,” and other symbols are pasted on the walls of the new home and the room of the newlyweds, among other things. On the wedding bed, dowry, wedding cake, and the table covered with “mandarin ducks playing in the water,” “butterflies love flowers,” and other red paper cuttings to express happiness and beauty, as well as the good wishes of many children and many blessings, the Hakka people enjoy putting paper cutouts of “Shao,” “Fu,” “Lu,” “Cai,” and other red paper cuttings on the door frames and walls, as well as paper cutouts. In some festivals, paper-cutting is merged with other art forms like lamps, dragon boats, paper-tying, printing, and dyeing, demonstrating strong practicality and decoration, which not only meets the aesthetic requirement but also serves the psychological demands of the participants.

### 3.3. Formal Beauty Is a Term Used to Describe the Appearance of a Person in a Formal Setting

When it comes to Gannan Hakka paper-cutting, the primary parts of the picture are dots, lines, and surfaces, which are used to communicate the main theme of the picture, as well as emotion and interest. The real and imaginary are interspersed, and a strong sense of rhythm and rhyme is demonstrated. More contrast, symmetry, and proportion, as well as other elements of beauty, should be incorporated into compositions. In the paper-cutting of Hakka dwellings, shown in Figure 3, the form of left and right symmetry is used, and the change of local patterns enhances the contrast effect in the picture, making the picture richer and more beautiful, reflecting the unique architectural characteristics and a complete and harmonious picture of life, as shown in Figure 3.

### 3.4. The Aesthetic Value of Ornamentation

The art of Hakka paper-cutting is a treasure trove of techniques that can be performed singly or in groups using various cutting, carving, tearing, and other technical methods. Clear outlines, smooth lines, and continuous qualities characterize paper-cutting patterns; delicate and sharp local patterns and details can be created with paper-carving, while irregular edges and natural texture effects characterize paper-tearing patterns. The image is exaggerated, full of variations, unified in color, simple, and concise, and the local decorative figures work together to create a pleasing composition. Overall layout is primarily based on the approach of scattered perspective, emphasize the corresponding virtual and real, full but not crowded, and uninterrupted, in order to create a generic, decorative artistic image. Examples include the work of the folk artist Zeng Xiaomei, who cut paper patterns, blending the image of people with popular auspicious patterns and words, resulting in a delicate and complete picture as well as engaging life scenarios.

### 3.5. Color and Beautification

The Gannan Hakka paper-cutting is influenced by the traditional Chinese color concept, the subjective consciousness of the creator, and the local cultural history. The application of color is symbolic, subjective, and associative in the Gannan Hakka paper-cutting. The majority of Gannan Hakka paper cuts are predominantly red, with contrasting colors, creating a powerful visual impression while also evoking the emotional traits of redness and festivity in the viewer. The visual and sensual perception of art is not only a reflection of humanity and emotion but also a reflection of human and sensory perceptions. “Expression through color” can be achieved through the use of paper-cutting, which not only reflects the attractive aesthetic impact but also conveys the emotion associated with the packing.

Because of the rich and diverse modeling contours, delicate and meticulous cutting techniques, simple and rustic content ideas, novel picture ideas, and extensive Hakka customs developed by Gannan Hakka paper-cutting, the art form has developed its own distinctive artistic style with strong aesthetic and application values. It is possible to beautify the packaging of local specialties by incorporating rich Hakka culture through paper-cutting art. This can help to strengthen the main image of the product, highlight the personalized characteristics of the product, and make the packaging design more aesthetic, emotional, and interesting. It also has a significant practical value. Meanwhile, it plays an essential role in the dissemination of regional culture, the promotion of regional economic growth, and the realization of economic value.

## 4. Digital Modeling and Visual Presentation of Paper Cuttings

### 4.1. Overview of Digital Modeling

As illustrated in Figure 4, the digital model of the paper-cutting pattern suggested in this paper is organized in a tree-like structure. A paper-cutting is composed of four layers: a top layer that contains the outer contour of the whole figure as well as all of its internal pattern elements, a second layer that is constructed by a variety of pattern elements according to a specific spatial distribution law and is used to describe the spatial construction pattern of the paper-cutting, a third layer that is constructed by a variety of similar pattern elements and used to describe the similarity between the two patterns, and the fourth floor is made up of various constructs. On the bottom layer, there is an element layer, which serves as a fundamental component of the entire paper-cutting and is formed as a result of the complete deconstruction of the previous layer.

This paper proposes a bottom-up kirigami structural pattern space analysis method for constructing the above-mentioned digital models. Firstly, the boundary pixels of the scanned paper-cut image are extracted, then each paper-cut pattern is obtained through preprocessing such as denoising and vectorization, and the element layer is constructed. For the purpose of clustering to obtain similar layers, it is necessary to construct a spatial distribution layer to detect the spatial distribution of the same type of kirigami patterns.

### 4.2. Preprocessing

The acquisition process of photographing and scanning introduces a large amount of noise into the paper-cut image, which is firstly preprocessed by median filtering with a filter window length of 3; then, the bitmap after filtering is used as the input, and the pixels with large differences in color from the 4 neighboring pixels are selected as the boundary pixels of the map; finally, these boundary pixels are traversed clockwise until they return to the starting point, and a closed sequence of boundary points is obtained, which is called a pattern element, denoted as

(1) $$\begin{array}{c} \left\{p_{i}\right\},i\in \left[0,m\right],p_{0}=p_{m}. \end{array}$$

A series of pattern elements are obtained by traversing all the boundary pixels of a paper-cut image, but they often contain too much detail, display poorly, store large amounts, and are not conducive to later editing. For this reason, in this paper, the boundary points of these pattern elements are fitted using cubic spline segments. First, the curvature value is calculated for each boundary point as

(2) $$\begin{array}{c} c_{i}=\frac{\left(p_{i-\delta }-p_{i}\right)\left(p_{i+\delta }-p_{i}\right)}{\left\|p_{i-\delta }-p\right\|\cdot \left\|p_{i+\delta }-p_{i}\right\|}, \end{array}$$

where the sampling interval *δ* is used to control the scale of this curvature, and this paper takes *δ*=5 [7, 20]. Then, take the local extreme points of curvature as key points; if the distance between the extreme points is too large, add key points appropriately, and get the key point sequence as

(3) $$\begin{array}{c} \left\{p_{i}^{*}\right\},i\in \left[0,n\right],p_{0}=p_{n}. \end{array}$$

Finally, the path between all adjacent key points *p*_*i*_^*∗*^ and *p*_*i*+1_^*∗*^ is fitted with the cubic spline, the boundary points on the path are sampled, the cubic spline is

(4) $$\begin{array}{c} f\left(t\right)=\sum_{i=0}^{3}f_{i}\cdot t^{i}, \end{array}$$

and the parameter *f* of cubic splines is calculated by minimizing the error of equation (5) [22, 23]:

(5) $$\begin{array}{c} \sum_{p_{j}=p_{i}^{*}}^{p_{j}=p_{i+!}^{*}}{\left[f\left(\frac{j}{l}\right)-p_{j}\right]}^{2}, \end{array}$$

where *l* is the number of sampled points on the path.

### 4.3. Similarity Analysis of Pattern Elements

To detect whether there is a similarity among the pattern elements in paper cutouts, this paper first calculates the matching error among the pattern elements using shape context descriptors and then clusters the similarity using spectral clustering. This method combines global shape context and local shape context descriptors, which overcomes the limitation that existing similarity calculation methods can only handle vector shapes with very consistent contours.

The matching error between each key point *p*^*∗*^ in element *C*_*a*_ of the graph and the key point *q*^*∗*^ in the pattern element *C*_*b*_ is defined as

(6) $$\begin{array}{c} E\left(p^{*},q^{*}\right)=\sum_{j=1}^{3}\sum_{k=1}^{8}\frac{{\left[h\left(p^{*},j,k\right)+h\left(q^{*},j,k\right)\right]}^{2}}{2\left(h\left(p^{*},j,k\right)+h\left(q^{*},j,k\right)\right)}. \end{array}$$

And the matching error of pattern element *C*_*a*_ with pattern element *C*_*b*_ is

(7) $$\begin{array}{c} E\left(C_{a},C_{b}\right)=\sum_{i=0}^{n-1}E\left(p_{i}^{*},q_{t}^{*}\right), \end{array}$$

where *t*=arg min_*j*_*E*(*p*_*i*_^*∗*^, *q*_*t*_^*∗*^).

Based on the matching error between two pattern elements, this paper divides them into several similar pattern element classes by the spectral clustering method so as to complete the construction of the similarity layer. First, we calculate the weight adjacency matrix *W*_*N*×*N*_ , which is

(8) $$\begin{array}{c} W\left(i,j\right)=\exp\left(-5\cdot \min\left(E\left(C_{i},C_{j}\right),E\left(C_{j},C_{i}\right)\right)\right). \end{array}$$

Use equation (8) in the weight matrix to calculate the nonnormalized Laplace matrix, which is

(9) $$\begin{array}{c} L=D-W. \end{array}$$

Then, the matrix *L* is analyzed for eigenvalues and *n* representative eigenvectors are obtained. Finally, *k*-means clustering is performed on these representative eigenvectors to cluster the pattern elements represented by them into *k*_*c*_ classes. In this paper, *k*_*c*_ is one of the parameters of this method, *k* is the parameter of spectral clustering, and based on the experimental effect, we set $\hat{k}=k_{c}$.

Existing paper-cutting digitization models represent paper-cutting graphics as a single-layer collection of many independent pattern elements, which can support efficient drawing but cannot meet efficient user editing. Even if the pattern elements repeat each other or are combined as a whole, users still need to edit them individually, which is not only time-consuming but also difficult to ensure the consistency of the editing effect. The digital modeling in this paper establishes a tree hierarchy according to the similarity of pattern elements and the spatial structure of the pattern so that the editing operation of a single pattern element can be transferred to other pattern elements of the same kind or the same pattern in real time, which saves the interaction time and ensures the consistency of the editing effect.

Based on the above digitization model, this paper develops an intelligent visualization tool based on computer graphics algorithms for existing paper-cut scanned images, including overall editing, local deformation, regularization, and visualization. These intelligent editing tools take full advantage of the three major spatial construction features of paper cutouts and can automatically migrate the interactive editing operations of a single pattern element to other pattern elements in the same similar class or motif. In addition, a paper-cutting design system based on shape retrieval was developed to quickly retrieve existing paper-cutting pattern elements and motifs based on user input of shape brushes and trajectory brushes. The simulation results are shown in Figures 5–8.

The first intelligent editing tools developed in this paper are the overall editing tools for paper-cut patterns, including panning, rotating, and scaling. They make full use of the log-polar frame computed from the global shape context descriptors, including the center point *o*, the principal direction *v*, and the radius size *R*, which are represented by the blue dots and the direction and the length of the green lines in Figures 5(c), 6(c), 7(c), and 8(c), respectively. In addition, the yellow arcs in these figures indicate the spatial distribution pattern trajectory lines of the pattern, while Figures 5(b), 6(b), and 8(b) visualize the corresponding tree hierarchy. The user drags the two endpoints of the green lines to complete any overall editing of one of the pattern elements, and the method in this paper automatically migrates the editing effect to other similar pattern elements in the same pattern or similar layers.  Figure 5 shows the intelligent overall editing of a paper-cut pattern composed of three different pattern elements, where the willow leaf pattern is rotated and dispersed, and the crescent serrated pattern is clustered.  Figure 6(d) shows the petal completion function of this paper, while Figure 6 shows the quick adjustment of the number of petals by the smart overall editing tool.

## 5. Conclusion

This paper proposes to develop a visual display system of Hakka paper-cut works in southern Gansu based on computer graphics algorithm. It also includes intelligent paper-cut functions such as translation, rotation, and zoom. Firstly, we calculate the similarity between pattern elements and cluster the vectorized independent pattern elements using the improved shape context descriptor. Then, the spatial distribution patterns of similar pattern elements are detected using the spatial distribution characteristics of traditional kirigami patterns. Furthermore, we employ a tree-like recurrent neural network to detect the spatial distribution patterns of similar pattern elements. Finally, a tree hierarchy is used to rapidly determine the system's overall geometric connectivity. Due to the spatial analysis of the aforementioned construction patterns, we automatically convert the input paper-cut into a tree hierarchy with four levels of root node, pattern layer, similarity layer, and element layer to complete the input paper-digital cut's modeling. Numerous experimental analyses demonstrate this method's effectiveness.

## Figures and Tables

**Figure 1:** Hakka folk paper-cut.

**Figure 2:** Hakka folk paper-cut.

**Figure 3:** Hakka folk paper-cut.

**Figure 4:** Schematic diagram of the paper-cutting hierarchy representation model.

**Figure 5:** The intelligent overall editing effect of this paper. (a) Input paper-cut images. (b) Digital mode visualization. (c) Local frames and patterns. (d) Intelligent visualization.

**Figure 6:** The pattern completion and quantity adjustment functions of the smart overall editing tool in this paper. (a) Input paper-cut images. (b) Digital mode visualization. (c) Local frames and patterns. (d) Intelligent visualization 1. (e) Intelligent visualization 2.

**Figure 7:** Smart local deformation effect of this paper. (a) Input paper-cut images. (b) Similarity clustering. (c) Local frames and patterns. (d) Intelligent visualization.

**Figure 8:** Shape regularity control tool. (a) Input paper-cut images. (b) Digital mode visualization. (c) Original image. (d) Complete regularization. (e) Semiregularization. (f) Antiregularization.

## Data Availability

The data used to support the findings of this study are available from the corresponding author upon request.
